The article "The Influence of Enterprise Culture Innovation on Organizational Knowledge Creation and Innovation under the Ecological Environment" was published in 2022. Journal: J Environ Public Health.

# The Influence of Enterprise Culture Innovation on Organizational Knowledge Creation and Innovation under the Ecological Environment

**DOI:** 10.1155/2022/3419918

**Published:** 2022-07-13

**Authors:** Ying Yuan, Tong Chen

**Affiliations:** ^1^College of Management and Economics, Tianjin University, Tianjin 300000, China; ^2^College of Management and Economics, Qinghai National University, Xining 810000, China

## Abstract

With the continuous development of economy and society, ecological environmental governance has been put on the priority agenda. In the process of ecological environmental governance, the state, society, and enterprises bear different responsibilities, respectively. As the main body of social economy, in the development of enterprises, the protection of ecological environment is the due meaning of enterprise culture is always paid attention. Whether enterprises can achieve success is not only directly affected by the development strategy, management mode, business philosophy, management tools, and other aspects but also indirectly affected by its own cultural construction level. Although corporate culture has changed due to the development of the network environment, the challenges of corporate culture innovation in terms of values and cultural conflicts should not be underestimated. It can not only enhance the centripetal force of all the employees but also enhance the competitive advantage of the enterprise. In addition, corporate culture also plays a positive role in enhancing office efficiency and increasing production capacity and output. Starting from the role of corporate culture, this study studies the characteristics of corporate culture under the background of implementing ecological environmental governance, addresses the challenges of corporate culture innovation in the new environment, and puts forward the measures of corporate cultural innovation, which provides reference for corporate culture innovation.

## 1. Introduction

The ecological crisis of globalization is an indisputable fact, China's situation is not optimistic, which makes our country ecological environmental management on the priority agenda ecological environmental management a complex system engineering, must adhere to the morality, the rule of law, and science and technology, therefore must strengthen bear responsibility, and build a reasonable and complete responsibility. In ecological and environmental governance, the government, enterprises, and other social organizations each perform their respective duties and assume their own responsibilities.

Ecological environmental governance refers to the establishment of a series of ecological environmental cooperative relations by various public or private institutions and managing ecological and environmental issues from different levels through the formulation and basis of certain norms and norms, to improve the ecological environment and promote sustainable human survival and development. As the main participant in the market economy, enterprises play an indispensable role in the ecological environmental governance. The responsibility of ecological and environmental governance and environmental protection should always be tied to enterprise status, reputation, development, and even life and death and can always be subject to social inspection and torture. Cultural factors are the indispensable basis and conditions for analyzing the operation of an enterprise, and corporate culture contains the social capital required for enterprise innovation. Enterprise innovation in the network environment is more dependent on enterprises to build high-quality modern social capital, and the construction of modern social capital that is compatible with enterprise innovation in the network environment is inseparable from corporate culture innovation [1]. High-quality modern social capital is an effective guarantee for the innovation of Chinese enterprises and an important means to improve the performance of enterprises.

In the process of continuous social and economic development, corporate culture plays an increasingly important role, and the construction of corporate culture is listed as an important part of enterprise development. With the deepening of market competition, enterprise management innovation has become inevitable, and only continuous innovation can improve their management quality and efficiency, thereby improving management advantages and promoting the sustainable development of enterprises. In the construction of corporate culture, publicizing corporate culture and transmitting corporate culture are an important way to reflect corporate values and development concepts. In addition, the construction of corporate culture can stimulate the creativity of employees, improve the efficiency of enterprise management, and ultimately complete the strategic development goals of enterprises. The development of modern enterprises, only through continuous innovation and upgrading, can maintain the same direction with the development of the times and add impetus to the development of enterprises. As the spiritual pillar of enterprise development, the innovation of corporate culture is the concept and viewpoint that enterprises break away from the previous cultural construction that are inconsistent with enterprise management and coordinate and match the development of enterprises with the environment, to form a culture that reflects corporate values. The relationship between corporate culture innovation and enterprise management innovation is very close, and it is necessary to face up to the relationship between the two, explore the important impact of corporate culture innovation on enterprise management innovation, and promote the vigorous development of enterprises.

Under the conditions of market economy in the information network era, with the continuous development of China's economy and society, how to innovate and shape corporate culture will attract much attention. The survival and development of enterprises are increasingly manifested as innovation and development of corporate culture, and the role of corporate culture in the survival and development of enterprises is becoming more and more important, which has become the cornerstone of enterprise market competitiveness and the key to determining the rise and fall of enterprises [2]. In the context of economic globalization and ecological and environmental governance, the innovative research of corporate culture should be based on a comprehensive, dynamic, historical, and global strategic vision, actively create a people-oriented, innovation-based corporate culture, and provide a strong and long-term strategic competitive development platform for the strategic development of enterprise management and scientific management. At present, corporate culture is the most ambiguous place in enterprise management, and it is also the most challenging link. The innovation and development of corporate culture have given modern enterprise management a new strategic significance.

## 2. Corporate Culture

### 2.1. The Concept of Corporate Culture

Corporate culture is a cultural phenomenon, which is formed in the operation and management process of enterprises. Corporate culture is the glue of employee values, moral codes, and behavior patterns and is a comprehensive reflection of the overall style of employees within the enterprise [3]. Corporate culture is also the embodiment of the core ideas of enterprise owners, with the help of cultural factors to form an impact on the work behavior, ideas, attitudes, and other aspects of internal employees and finally form a holistic cultural atmosphere through continuous accumulation [4]. Once the corporate culture is completed, the role played by its own operation and management cannot be underestimated. Corporate culture is formed on the basis of the core value system of the enterprise, with a continuous common cognitive system and habitual behavior. The structure of corporate culture is divided into four levels: the core layer (values), the deep layer (behavior level), the institutional level, and the image level [5], as shown in Figure 1.

Corporate culture is the organizational culture of the enterprise, which revolves around all aspects of enterprise operation and management. The management of the enterprise is inseparable from the enterprise team spirit, corporate culture has a positive impact on the creation of corporate team spirit, the team responsibility awareness, and the sense of mission to improve the role of promotion and can be understood as all internal employee codes of conduct and values of the unified performance, and the employee behavior has a positive incentive effect and can make active participation in corporate activities, for the enterprise to make more contributions. As shown in the figure, the content of corporate culture mainly includes three dimensions: innovative values, innovative systems, and behavior patterns [6], as shown in Figure 2.

With the continuous development of social economy, people constantly plunder natural resources and the discharge of various toxic and harmful substances. Today, ecological and environmental governance has become a major event concerning the rise and fall of the world. Under the background of the current development of our national ecological civilization, only when enterprises can constantly improve their own mechanism and constantly strengthen the quality of environmental management in the enterprise culture, they can promote the sustainable and stable development of enterprises. In this context, the model of enterprise culture construction also needs to be innovated.

### 2.2. The Role of Corporate Culture

The value of corporate culture is mainly reflected in the needs of self-interest, through observing the changes in the ideology and spiritual atmosphere of internal employees, with the help of reasonable guidance means to gradually cultivate the value concept that caters to the development and business objectives of the enterprise [7]. As shown in the figure, corporate culture plays a central role in the construction of the company and can unite all aspects of the company's construction, as shown in Figure 3.

#### 2.2.1. Guiding Role

The formation of corporate culture is based on the premise that the values, interests, and management concepts of enterprise employees are consistent with each other. Corporate culture has a guiding function, and it can clarify the development goals and directions for the enterprise, enhance the fit of employee behavior and corporate culture, let employees decide their own words and deeds according to the development goals and development direction of the enterprise, and not only can enhance the self-discipline of their own behavior but also an effective way to motivate employees' enthusiasm [8].

#### 2.2.2. Incentive Effect

This incentive effect is mainly reflected in two levels: one is the spiritual level of employees and the other is the material level of employees [9]. Whether the corporate culture is excellent is directly related to the degree to which the employees of the enterprise improve their comprehensive ability and quality and also determines the degree of contribution of each employee to the development of the enterprise. In the process of building corporate culture, it must closely focus on the core concept of being people-oriented, paying attention to respect, trust, and care for people, and helping employees to achieve role transposition, from the hired subject to the ownership of the enterprise, so that it is more conducive to tapping the potential value of employees and contributing more youth and enthusiasm to the enterprise.

#### 2.2.3. Binding Effect

This constraint is not mandatory, but achieves the restraining effect of implicit influence through the subtle form. If an employee's words and deeds are contrary to the corporate culture, it will inevitably be rejected by other employees, and this invisible pressure will inevitably change the wrong words and deeds of employees for a long time, enhance self-discipline, and reintegrate into the collective to work together for the development and progress of the enterprise.

#### 2.2.4. Cohesion

The formation of corporate culture helps to enhance the connection between the main body of the enterprise and the internal employees, and employees can continuously improve themselves while the enterprise obtains rapid development. Looking at the cultural construction of major outstanding enterprises, “cohesion” is the focus of emphasis. Generally speaking, the development of enterprises needs three ties (cultural ties, power ties, and capital ties) as the bridging point for each factor of production, and the role played by the Chinese ties is the most important [10].

#### 2.2.5. Radiation Effect

In addition to the above four functions, excellent corporate culture can also play an important role in social opinion. The evaluation of the external image of the enterprise by all sectors of society also determines the competitive strength of the enterprise in a certain aspect. Based on the Internet age, there are many carrier tools that can be relied on to exert the radiation effect of culture, such as communication media and public relations.

### 2.3. Characteristics of Corporate Culture

Corporate culture is abstract. In the networked society, the culture of each enterprise is unique and has a binding role. In the process of building corporate culture, managers develop relevant strategies and rely on the transmission mechanism of the information platform to let employees understand the business objectives and business direction of [11]. The specific arrangements of various affairs of the enterprise are also realized by relying on the various functions of the network platform and the corporate culture formed by employees through the integration with corporate values; on the contrary, the values expressed in the corporate culture are also transmitted and shared among employees, thereby enhancing the sense of belonging and honor and disgrace of employees to the enterprise.

In the network society, the focus of enterprise management has also undergone great changes, mainly manifested in the transformation from groups to unit individuals. In this context, traditional rules and regulations are gradually being replaced by online platform information, and the corresponding managers' rights and decisions have also been weakened [12]. Therefore, the management of modern enterprises can no longer follow the previous centralized management model, but needs to be converted to a decentralized management model, through the construction of corporate culture to standardize internal governance and enhance the degree of compatibility between individual employee behavior and the overall development goals, which is also a necessary premise for the long-term survival and development of enterprises.

Because the Internet has the characteristics of fast information dissemination speed and wide dissemination range, it greatly enhances the penetration ability of corporate culture, and the information between the senior management of the enterprise and ordinary employees can be quickly disseminated and interacted in a timely manner. In the network environment, enterprises should regard interactive culture as the key core of cultural construction, and the emergence of network technology has enabled culture to be shared and broken through the hierarchical barriers due to the previous internal structure [13]. Don in the book “Digital Growth” published by Tapsco mentioned that in the network each individual is not only a participant in culture but also a maker of culture, and the original intention of network culture is to carry out a virtuous circle among network users by completing the construction of information transmission bonds. It can be seen that if you want to do a good job in building and maintaining network culture, you need the joint efforts of all participants, and relying solely on information technology will not work [14], as shown in Figure 4.

As shown in the figure, Denison's organizational culture evaluation model, he completed the construction of the organizational culture model on the basis of the corporate culture scale. The model is highly applicable, which can not only reflect the connection between the stability and flexibility of the enterprise but also reflect the internal and external concerns of the enterprise. He also analyzed the effectiveness of corporate culture and corporate organization from four levels (consistency, mission, adaptability, and participation), and on this basis, he divided the evaluation model structure into 12 specific aspects [15]. As can be seen from the above figure, the two cultural characteristics on the left and the right, respectively, reflect the flexibility, change, and stability of the enterprise. The two cultural characteristics of the upper and lower levels reflect the external and internal concerns of the enterprise.

Participation: the evaluation scope of this dimension includes the sense of responsibility, business performance, and ownership psychology of enterprise employees, and according to the questionnaire analysis structure, it can reflect three aspects of enterprise employees: 1. employee ability; 2. close communication; and 3. trust in authorization and ability [16]. There are three indicators involved, namely indicator 1 (authorization), indicator 2 (team positioning), and indicator 3 (capacity improvement). There are many factors that can be reflected in the authorization indicators, such as the intensity of employees' sense of belonging to the company and their positive attitude towards their own work. The elements reflected in team positioning indicators include the degree of importance that enterprises attach to employees' cooperative behavior and the degree of dependence of employees on teams when carrying out specific work. Elements that reflect competency improvement indicators include the importance that companies attach to employee training and the performance of employees' need to learn new knowledge.

Consistency: the evaluation direction of this dimension mainly focuses on two aspects: one is to reflect the performance of the internal culture of the enterprise in the strength of cohesion and the other is to reflect the current situation and value of the core culture construction. This dimension examines three aspects of the enterprise: the first is core values, the second is internal consensus, and the last is coordination. Elements reflect core values, such as whether all employees of the company have common values or the degree to which the employees of the company recognize these values. On the representative elements of internal consensus, such as whether the leadership of the company's senior management can make subordinate employees converge in various aspects, and on some core interest issues, employees, leaders, and enterprises can reach consensus. The elements reflected in the indicators of harmonization include whether the internal levels and departmental agencies of the enterprise are more complex and whether there is a strong cooperative relationship between various departments.

Mission: this dimension is the ultimate reflection of the long-term interests of enterprises and the emphasis on development planning, and it can be divided into three subdimensions, namely indicator 7 (vision), indicator 8 (strategic goal), and indicator 9 (strategic orientation). As far as the vision indicators are concerned, they mainly reflect two points: one is the degree of expectation of enterprise employees to the main body of the enterprise; the other is the acceptance of expectations by enterprise employees, for example, the sense of consensus shown by the employees of the enterprise on the future scenarios of the enterprise and whether the employees can fully agree with and accept this vision. As far as strategic orientation is concerned, it is mainly a reflection of the strategic willingness of the enterprise, such as the level of competitive goals in the industry in which the enterprise is located and the depth of the perception of the strategic orientation of the enterprise by the employees of the enterprise. Strategic goal indicators are mainly a concrete reflection of strategic orientation, for example, whether the enterprise has formulated in detail in terms of development planning and whether it decomposes the overall goal of the strategic plan and then passes it on to each employee layer by layer as a specific reference for carrying out the work.

Adaptability: the evaluation scope of this dimension mainly focuses on two aspects: the first is the sensitivity of the main body of the enterprise when the external environmental changes; the second is the ability to cope with the external dynamic environment. There are three indicators involved, namely indicator 10 (organizational learning), indicator 11 (customer first), and indicator 12 (innovation and change). Organizational learning indicators mainly reflect the ability of enterprises to respond to changes in the external environment, such as whether the company continues to innovate internal aspects around changes in customer needs and whether it can cater to changes in the market environment to carry out new knowledge acquisition training for employees. The indicators of creating change mainly reflect the attitude of enterprises in the use of innovation factors, such as whether enterprises are willing to accept various risk losses caused by innovative changes and the ability of enterprises to change as the external environmental changes. Customer first indicators mainly refer to the service attitude of enterprises to customers, for example, whether the enterprise can use customer needs as an entry point to analyze customers in combination with the external environment and enhance the customer's sense of experience and satisfaction and whether the enterprise has a certain perceived omen when customer needs change.

### 2.4. The Concept and Concept of Corporate Culture Innovation

#### 2.4.1. The Concept of Corporate Culture Innovation

Corporate culture innovation is mainly reflected in two aspects, namely the innovation of concepts and the innovation of the system, and corporate culture innovation occupies an important position in enterprise management and is the foundation of enterprises to maintain strong vitality, but also an important accumulation process of enterprise spiritual wealth. Through corporate culture innovation, enterprises can form a unique style, thereby highlighting the maximum advantages of enterprises.

#### 2.4.2. The Role of Corporate Culture Innovation

Although corporate culture innovation cannot directly bring economic income and material wealth to enterprises, the wealth it brings will be reflected in other forms. From the perspective of the long-term development of the enterprise, the wealth brought by the corporate culture is priceless, and it will exert greater value with the development of the enterprise, and it is also visible that the economic benefits cannot be replaced. Corporate culture is equivalent to national culture; for a nation, national culture has a unique charm, in the long river of history to play a huge role in the development of the river. Corporate culture, as the spiritual pillar and spiritual wealth of enterprise development, must be based on the development of the enterprise itself in the process of innovation and shape a culture that highlights the characteristics of the enterprise. In the process of corporate culture innovation, it is necessary to continuously guide enterprise employees to attach importance to cultural innovation, closely link enterprise innovation with personal development, and continuously improve the centripetal force of enterprises. From the perspective of the internal level of the enterprise, the innovation of corporate culture is conducive to the improvement of corporate image and influence and is conducive to the shaping of corporate brand. Through corporate culture innovation, enterprises can face up to their own development more squarely, lock the course in development, and continue to move in the right direction.

## 3. The Innovation of Corporate Culture in the Ecological Environment

With the increasing requirements of the society for the ecological environment, enterprises assume more due to social responsibilities. The importance of enterprises to the ecological environment also greatly affects the production operation and production management of enterprises. The production efficiency and operational efficiency of an enterprise depend on the enterprise culture, and to improve the management quality and competitiveness of the enterprise, it is necessary to continuously innovate the enterprise culture in the network environment [17].

### 3.1. Environmental Management Mechanism in Corporate Culture

Enterprise environmental management mechanism refers to the enterprise according to the current social sustainable and stable development; in the process of enterprise management of an ecological environmental protection concept, from the current management in the process of multiple links to control pollution, through this form of resource resources, it finally achieves enterprise economic benefit and corporate social benefits and environmental protection benefits between efficient unified management form and operation mechanism. As shown in Figure 5, there are three different levels of the current enterprise environmental management mechanism: at the macro-level, an industrial environmental management system is the development body, at the micro-level, and the public and NGOs. In addition, some scholars put forward that the current enterprise environmental management form mainly involves four different modes, the current enterprise environmental management committee, and environmental protection professional functional departments of the mutual integration of a management form and ISO14000 management mode. So, we can conclude that the development of the current environmental management system is a diversified structure management system, itself is through the international community and governments, enterprises, nongovernmental organizations, and the public participation, mainly through ecological ethics and environmental system, social development mode and human survival concept and mode, ecological culture education, ecological technology development and application level and enterprise management, and many different factors; the ultimate purpose is to promote the current enterprise resource-saving and environmentally friendly enterprise goals of a management form and specific operation mechanism.

Under the premise of more perfect environmental management mechanism, the ideology, values, and behavior methods of employees have also undergone profound changes, and the enterprise is faced with many new problems and new challenges. The following table shows the measurement scale of corporate innovation culture. It can be measured through the three dimensions of innovation values, incentive system, and behavior mode, to obtain the new challenges faced by corporate culture in the ecological environment. Tables 1 and 2 are the summary data for the valid samples of the questionnaire design survey.

As the endogenous driving force of enterprise innovation, innovation culture can lead all employees of the organization to work together to create an innovation blueprint, and the strong atmosphere of innovation culture helps to promote the innovation performance of enterprises [18]. Figures 6 and 7 show the analysis of the influencing factors of innovation culture on corporate performance in the study and the analysis of the impact path. The path coefficients of enterprise innovation values, incentive systems, and behavior patterns to innovation performance are 0.51, 0.50, and 0.37, respectively, indicating that there is a significant positive correlation; that is, innovation culture and innovation performance are positively correlated. Cultural innovation ability reflects the innovation competitiveness of enterprises, the strength of innovation ability directly affects the innovation status and honor of enterprises in the market, high innovation ability is often accompanied by high market acumen, reaction ability, resource integration ability, resource utilization efficiency, financial level, and finally comprehensive performance of enterprise innovation performance. The stronger the excellent innovation culture, the greater the enthusiasm and enthusiasm of all employees to innovate, the stronger the learning and practical ability, and the faster the new ideas are generated and transformed, and these positive effects will eventually cultivate high innovation ability.

### 3.2. The New Phenomenon of Enterprise Culture under the Ecological Environment

#### 3.2.1. The Value of the Enterprise as a Whole Is Supreme, and the Values of Suppressing Individuality Are Challenged

The values of traditional enterprises that emphasize the overall interests and ignore the individual interests are greatly challenged.  Figure 8 shows the results of an evaluation of the core values of an enterprise. From the result, it is not difficult to conclude that the corporate culture has formed a “decentralized,” people-centered, and individual-centered pattern, and the pursuit of equal interaction and mutual benefit culture has become the trend of The Times. Enterprises must change the traditional hierarchy, administrative management bureaucratic management mode, and users' zero distance interaction [19]. Only by changing the way of thinking and business philosophy of enterprises we can adapt to the changes in the environment.

The emergence of the mobile Internet has made changes in the way enterprises operate and manage, free WeChat has robbed China Mobile, Unicom, and Telecom of their jobs, DiDi Taxi has disrupted the taxi industry, and Yu'e Bao has absorbed 57.1 billion yuan in deposits in 18 days, robbing state-owned commercial banks. The rapid development of mobile Internet has promoted the cross-border operation of the industry and the integration of resources, and the competitive environment has become more complex, and new technologies such as mobile Internet, big data, O2O, Industry 4.0, new energy, new materials, environmental protection, and energy conservation are changing the original economy and commerce. The pattern has an important impact on the way of thinking, behavior, life, and work of enterprise employees, especially young employees. The values of traditional enterprises that emphasize the interests of the whole and ignore the interests of individuals have been greatly challenged, and the following figure shows the results of an evaluation of the core values of a company. From the results, it is not difficult to conclude that corporate culture has formed a pattern of decentralization, people-centered and individual-centered, and the pursuit of equal interaction, mutual benefit, and win-win culture has become the trend of the times. Enterprises must change the traditional hierarchical, administratively bureaucratic management model and interact with users at zero distance [19]. Only by changing the way of thinking and business philosophy of enterprises we can adapt to changes in the environment, as shown in Figure 8.

#### 3.2.2. The Relationship between the Government and Enterprises under the Background of Ecological Environmental Governance

Traditional ecological environmental governance takes the government as the main body, and enterprises are forced to implement relevant environmental protection policies. In the current social background, enterprises and governments and government show a trend of cooperative governance. The important difference between cooperative governance and traditional public administration is that it breaks the unity of the political objectives of public policy and separates policy from the linear relationship of the single line solely by the political institution. Under the condition of cooperative governance, the external function of administrative power will be greatly weakened, and the governance subject will no longer rely on the power to directly act on the governance object. The state of administrative power serving the abstract public interest will also change, which will be closely related to the moral consciousness of the holders of administrative power, which is the basic feature of cooperative governance [20].

In the process of ecological and environmental governance, the introduction of public-private partnership not only realizes the complementary advantages between the public and private sectors but also realizes the effective risk sharing. In this way, in the process of ecological and environmental governance, the advantages of the public and private sectors can be fully brought into play to play the effect of promoting strengths and circumventing weaknesses and achieving win-win cooperation. In terms of advantages in the process of environmental governance, the public sector makes use of its own advantages to formulate corresponding specific policies and establish strong policy support and administrative system, so that public projects can get strong support. However, in terms of ecological and environmental governance, the public sector is constrained by budgetary constraints and the lack of sufficient funds, which are often the constraints that cannot be ignored. In addition, the government lags behind enterprises in project management, and the government management efficiency is relatively low, which is a genetic defect in the public sector, and it is often difficult to overcome by itself.

The private sector, however, is relatively funded high management and competitive innovation mechanisms, but the disadvantage of the private sector is that it often faces greater risks and instability. If public-private partnerships are adopted in the environmental governance process, the public and private sectors can complement and complement each other. Public-private partnerships can not only contribute to ecological and environmental governance, but more importantly the competition mechanism in public-private partnerships can enable both parties to pay more attention to the quality of the public services provided. Competition makes the private sector in public-private cooperation more active in providing public services and improving the quality of services, which is conducive to achieving efficient ecological and environmental governance.

The relationship between the innovation and development of corporate culture and modern network, economy, society, humanities, and other aspects is correctly handled. Corporate culture is a management ideology and concept formed and developed on the basis of modern civilization, contemporary network informatization, and market economy globalization and is an integral part and embodiment of the core values of socialism. It is changing people's production and lifestyle, changing people's values and outlook on life, and injecting new vitality into the development of society and culture. Today's network information society is an era of great integration of modern cultures such as network, information, and knowledge, and the cultural literacy of enterprise managers directly affects the innovation and development of corporate culture. The innovation and development of corporate culture are a good embodiment of the survival and market competitiveness of enterprises.

## 4. The Network Environmental Corporate Culture Innovation Strategy

Under the conditions of market economy in the information network era, with the continuous development of China's economy and society, how to innovate and shape corporate culture will attract much attention. As an informal system of the enterprise, corporate culture can essentially shape the personality of the enterprise and the behavior of employees. The role of corporate culture in the survival and development of enterprises is becoming more and more important and has become the cornerstone of enterprise market competitiveness and the key to determining the rise and fall of [21]. Under the condition of economic globalization and information network, the innovation of enterprise culture research, to a comprehensive, dynamic, historical, and global strategic vision, actively builds people-oriented, innovative enterprise culture, the harmonious development of man and nature into the enterprise culture, for enterprise management strategy development and scientific management to provide strong and long-term strategic development platform, as shown in Figure 9.

The construction of traditional corporate culture mainly starts from the three aspects of spiritual culture (MIS), institutional culture (BIS), and visual culture (VIS) to shape the image of characteristic culture and promote the growth of enterprises [22], but under the requirement of sustainable development, enterprise culture needs to adapt to management and development, establish humanistic echo new culture innovation system, enterprise culture into two-way interactive communication, enterprise only change the thinking of enterprise culture construction, give full play to the role of new media, the media, enterprise internal, and external publicity, carry forward the enterprise culture tradition, strengthen the propaganda of environmental protection, and can really do well the enterprise culture construction and environmental protection mechanism construction.

### 4.1. Adhere to the People-Oriented Corporate Culture Concept

The purpose of corporate culture innovation is to improve the internal cohesion and external competitiveness of the enterprise, to promote the overall progress of the enterprise. The purpose of corporate culture innovation is to improve the internal cohesion and external competitiveness of the enterprise, to promote the overall progress of the enterprise. The fundamental factor of enterprise development is people, and people are also the most active factor in the productivity of an enterprise. The harmonious coexistence of people and environment is the inevitable of social development, and enterprise culture construction from the enterprise development strategy, according to the characteristics of flat and network organization, adheres to the people-oriented, through the joint efforts of all staff, creates positive cultural atmosphere, forms and meets the needs of the mainstream organization of enterprise values, and builds the spiritual culture of the enterprise. The culture of Alibaba subsidiaries has its own characteristics: Alibaba Company pursues steadiness and efficiency; Taobao culture is younger and more lively, close to grassroots, and Alipay and Yahoo are close to elite culture. As Zeng Ming, president of Yahoo China, said, “The best culture should match the corporate customers and the living environment they live.” Peter to network organization to a symphony orchestra, in the “symphony orchestra,” only one highest conductor, composed of organization members is a large number of experts, and they work in accordance with the unified “movement,” “conductor-musician,” and “musician-musician,” and the “instruction” between “communication” is the electronic pulse and network. Nowadays, because of its convenience, immediacy, and accuracy characteristics, the mobile Internet has penetrated into people's work, life, and entertainment and also promotes the reform of enterprise management. The creativity and enthusiasm of employees have become the core driving force for the survival and development of the enterprise. Therefore, managers need to give up the centralized control of the organization and adopt decentralized management to ensure the flexibility of the organization. At the same time, the corporate culture needs to maintain the effective operation of the organization, and people-oriented has become an inevitable requirement of the enterprise. Mr. Smith, the founder of FedEx, the world's largest express delivery company, said employees are an integral part of the decision-making system. “Putting people first, they provide a high level of service and profits follow.” Enterprise managers should pay attention to the changes in employees' demands, pay attention to the personal growth and physical and mental health of employees, especially the new generation, increase communication channels, build a platform for employees to show their talents, and enhance their sense of belonging.

Therefore, in the process of corporate culture innovation, we must always focus on the common values of the “two supremes” industry and combine the actual formation of our own unique cultural concepts, and in the process of practice of the implementation of business policies, strategies, etc., we must summarize the practical experience in a timely manner, upgrade it to a value concept recognized by all employees, and resolve the shortcomings of corporate culture package customization.

### 4.2. Formulate a Corporate Culture Landing System and Strengthen Execution

The management system of the enterprise can help the enterprise to pursue the greatest economic interests. The enterprise management system is a mandatory obligation formulated by an enterprise in the production and operation management activities, and the provisions or regulations that can guarantee certain rights cover all the rules and regulations of the enterprise, such as the personnel system, the production management system, and the democratic management system. One of the important components of corporate culture is the institutional culture of the enterprise, which is also the carrier and foundation of the spiritual culture of an enterprise. Excellent corporate culture is reflected in the scientific, perfect, and user management system and management methods. The construction of enterprise culture must ultimately be implemented in the system, and a standardized management system can be formed to make the behavior of enterprise employees have rules to follow, laws to follow, and avoid or reduce blindness in construction. The system is a strong guarantee for the landing of corporate culture, and a reasonable system culture has a good guiding, motivating, and restraining effect on the behavior of employees. It should be noted that when formulating a system or a system conflict or absence, the spirit of the corporate culture concept must be taken as the criterion to ensure the smooth implementation of the corporate culture. When a company's strategic objectives change significantly, the rules and regulations of the enterprise must change from time to time. At the same time, different employees under the network economy should be treated differently, such as repetitive work to adopt quota assessment and innovative work to adopt flexible system incentives; in-house is suitable for a clear division of labor, and fieldwork should be flexible and appropriately authorized. Alibaba's quarterly supervisors conduct behavioral assessments of each employee in two parts: performance and values account for 50% each. Each concept in the corporate culture value system must be supported and implemented by the corresponding management system, and the implementation of the system, the supervision of the subordinate to the superior, and the suggestions of employees are all included in the system design. This is conducive to breaking the backward management system, enabling employees to participate in management, and stimulating employees' enthusiasm and professionalism. According to the characteristics of networking and platformization in the Internet era, Haier has explored and established a “win-win-win model for people in one,” turning employees into entrepreneurs and becoming their OWN CEOs through employee customization The flat organization implements platform management and builds enterprise employees, suppliers, and users into a community of interests, thus forming a new enterprise ecosystem, truly making enterprises responsible for users, realizing seamless docking between enterprises and users, and turning the external coercion of corporate culture into an internal drive.

### 4.3. Innovation Builds the Enterprise Culture Material Layer

The material layer of corporate culture is the external layer of the core layer of corporate philosophy, the most basic content of corporate culture, as the visual part of the direct perception of the public inside and outside the enterprise, and also the basic basis for the public to evaluate corporate culture.

In the network environment, it is necessary to incorporate elements related to the corporate culture of “Internet +” and the grid into the corporate culture, as shown in Figure 10.

The material layer of corporate culture mainly includes four major systems of visual recognition, material environment, product matching, and cultural dissemination, and enterprises can put forward the planning and principles of material culture construction, hire professionals to complete specific business, and corporate culture management personnel participate in and supervise and check, mainly from four aspects:

First, comprehensive planning is implemented step by step. The construction of the material layer of corporate culture needs to be carried out in accordance with the principles of overall planning, inheritance, and innovation, and step by step, with high standards and strict requirements, and implemented step by step at different levels and in different professions, to display the corporate brand image and highlight the personality of corporate culture.

Second, the cultural environmental experience is enhanced. It is necessary to design an attractive cultural environment, attract employees to participate in, and strengthen the cultural experience through celebrations and cultural and sports activities, to achieve edutainment, create a lively corporate culture atmosphere of full co-construction, and infect, educate, and motivate employees with a good cultural environment.

Third, the carrier of corporate culture is improved. The material layer of traditional corporate culture construction continues to expand to all aspects of the enterprise supply chain and value chain, actively attracts corporate shareholders, customers, suppliers, and the public to participate in the construction of corporate culture, and improves the corporate culture system through two-way dissemination of culture, to shape a good corporate image.

Forth, in addition to the traditional carrier brand trademark, building environment, visual identity, and product packaging, we should also pay full attention to the construction of network carriers such as intranet, extranet, international Internet, WeChat, and Weibo. Various new media are fully used, and a variety of platforms to spread corporate culture are built, such as organizing brand promotion, customer friendship, employee recognition, and colorful cultural activities, enriching the spiritual and cultural life of employees, breaking the cold network relationship, promoting employees and enterprises to breathe together and share a common destiny, and stimulating employee team spirit. New media tools such as email, BBS, MSN, and QQ are fully used and be easily accepted by employees. The BBS of the enterprise can become the position of publicizing the corporate culture, and the employees can anonymously express their dissatisfaction with the enterprise, make suggestions and opinions, release the relevant information of the enterprise through the BBS, and carry forward the main theme of the corporate culture by correctly guiding and disseminating the corporate culture. For example, Huawei in Shenzhen uploads stories promoting the core values of the company to the BBS community, makes videos for employees to watch, and timely releases dynamic information about the enterprise, and the access rate is very high. As the main mobile device in the era of mobile Internet, enterprises need to use mobile phones to strengthen the implementation of corporate culture. Establish a mobile newspaper for corporate culture work, integrate corporate news, business knowledge, and other information, and publish it regularly through mobile phones, so that employees can participate in corporate culture work in a timely manner. By using the WeChat function of mobile phone, establish a WeChat communication platform for corporate culture, carry out various discussions, and realize the landing of corporate culture.

## 5. Conclusion

Under the condition of increasing social requirements for sustainable development, due to the social-ecological subject status of enterprises, the protection of ecological environment has brought new requirements to the management and management concept of enterprises. At the same time to the construction of enterprise culture and environmental protection mechanism brought new challenges, employees organization hierarchy concept, democratic consciousness, the pursuit of equality, and mutual benefit culture become irreversible trend, enterprise culture from one-way spread into two-way interactive communication and enterprise ecological environmental protection and management from passive to active. Therefore, in the context of ecological environmental governance, we must pay attention to the participation of corporate culture, give full play to the role of new media and we-media, adhere to the people-oriented corporate culture concept, actively publicize environmental protection policies and environmental awareness, pay close attention to green and sustainable development in the operation of enterprises, integrate ecological and environmental protection into the corporate culture gene, formulate the enterprise culture implementation system and strengthen the executive force, make full use of the various new media outlets, to build various platforms to spread corporate culture, carry forward the corporate culture and tradition, make employees timely participate in the corporate culture work, through “into the brain,” “into the ear,” and “into the heart” to achieve corporate culture landing, to achieve full participation of government, businesses, and individuals, and finally realize the improvement of the ecological environment is realized.

In summary, corporate culture innovation to a large extent affects the enterprise management innovation, and corporate culture innovation can continuously improve the centripetal force and cohesion of the enterprise, reflect the core values of the enterprise, play a positive guiding role in enterprise management innovation, point out the direction for it, improve the innovation and creativity within the enterprise, constantly promote the innovation and improvement of various management systems of the enterprise, and fundamentally improve the enthusiasm of the employees of the enterprise. Employees who engage in their work with a more proactive attitude will achieve more results with less effort. The formation of corporate culture is a slow process, and this process requires continuous reflection, breakthrough, abandonment, and sublimation, so that enterprises maintain inexhaustible power, to meet the challenges of the market with a better attitude. Therefore, through corporate culture innovation, enterprise management innovation can be realized, the operating efficiency of enterprises can be improved, and the maximum value of enterprises can be realized, to complete the long-term strategic development goals of enterprises.

## Figures and Tables

**Figure 1:** Four levels of corporate culture.

**Figure 2:** Three dimensions of corporate culture content.

**Figure 3:** Central role of corporate culture.

**Figure 4:** Denison organizational culture evaluation model.

**Figure 5:** Three levels of ecological environmental management system.

**Figure 6:** Innovative culture validation factor analysis model.

**Figure 7:** Path of influence of enterprise innovation culture on innovation performance.

**Figure 8:** Evaluation results of a company's core values.

**Figure 9:** Theoretical model of corporate culture innovation.

**Figure 10:** Integration path of corporate culture.

**Table 1:** Measuring scale of enterprise innovation culture.

Dimensionality	Title item	Variables
Innovative values	Encourage challenges to the status quo and try new ideas, new perspectives, and new methods in this position	XJ1
	Tolerate innovation failures and mistakes and do not punish them	XJ2
	Keeping promises and taking responsibility	XJ3
	Open communication channels and information-sharing channels	XJ4
	Employees have a lot of freedom to do what they are interested in	XJ5

Incentive system	Each department has a model innovator	XZ1
	Every successful innovation is rewarded	XZ2
	Each employee has an innovation target, and employees who fail to complete the innovation target should be appropriately punished and criticized	XZ3
	The company will regularly train all employees on innovative knowledge and skills	XZ4

Behavior patterns	Encourage diversified, multichannel, and multi-departmental learning from each other	XM1
	Encourage employees to share innovative projects, while the originator of the innovative idea can participate in the implementation process of the innovative project	XM2
	Dissent is considered a positive act of innovation	XM3

**Table 2:** Statistical table of sample structure of enterprise innovation culture survey.

		Frequency	Effective percentage
Number of years of business establishment	Less than 2 years	35	15.9
	2–5 years	72	32.7
	5–10 years	73	33.2
	More than 10 years	40	18.2

Number of employees	Less than 10 people	19	8.6
	10–100 people	85	38.6
	100–500 people	81	36.8
	500 and above	35	15.9

Age	Under 25 years	17	7.7
	26–35 years	97	44.1
	36–45 years	74	33.6
	46–55 years	25	11.4
	55 years and above	7	3.2

Number of years of work	Less than 3 years	19	8.6
	3–5 years	77	35.0
	5–10 years	69	31.4
	10–20 years	34	15.5
	20 years and above	21	9.5

Industry	Production	24	10.9
	Electronic information services	29	13.2
	Finance and insurance	55	25.0
	Commercial industry	28	12.7
	Education industry	41	18.6
	New energy industry	24	10.9
	Pharmaceutical industry	12	5.5
	Other	7	3.2
Total		220	100

## Data Availability

The labeled data set used to support the findings of this study is available from the corresponding author upon request.

## References

[1] Attah-Boakye R., Adams K., Kimani D., Ullah S. (2020). The impact of board gender diversity and national culture on corporate innovation: a multi-country analysis of multinational corporations operating in emerging economies. *Technological Forecasting and Social Change*.

[2] Assefa G., Kijora D., Kehaliew A., Bediye S., Peters K. J. (2020). Creativity and corporate culture. *SSRN Electronic Journal*.

[3] Chen C. H. (2022). *The Mediating Effect of Corporate Culture on the Relationship between Business Model Innovation and Corporate Social Responsibility: A Perspective from Small- and Medium-Sized Enterprises*.

[4] Danko T. P., Kazaryan M. A., Pervakova E. E., Novikov A. A., Novikova E. V., Sekerin V. D. (2018). Influence of corporate culture on the efficiency of innovation in russian companies. *International Journal of Civil Engineering & Technology*.

[5] Ellis R., Hong T. D., Roberts E. H. (2021). *Managing Value Co-creation in University-Industry Partnerships*.

[6] Feng G., Wang J. (2020). The impact of corporate social network on innovation: a mediation analysis of agency costs and financial constraints. *Journal of Mathematical Finance*.

[7] Hao-Qiang W. U., Economics S. O. (2019). Corporate culture and M&A technology innovation efficiency from the perspective of corporate property rights. *Journal of Finance and Economics Theory*.

[8] Hatanmaa (2018). *Induction to Innovation Culture: Case Study of Facilitating New Employee Innovativeness*.

[9] He M., Lee J. (2020). Social culture and innovation diffusion: a theoretically founded agent-based model. *Journal of Evolutionary Economics*.

[10] Jin H., Qianya P., Zhang G. (2019). *The Appearance of Research on the Relationship between Culture and Innovation*.

[11] HezewijkJnah A. J., Beem A. P. V., Verkleij J. A. C., Pieterse A. H. (2019). About face: toward a culture of innovation. *Canadian Journal of Botany*.

[12] MüllerKitchell S., Cooper E. J., Alsos I. G. (1995). Corporate culture, environmental adaptation, and innovation adoption: a qualitative/quantitative approach. *Journal of the Academy of Marketing Science*.

[13] Liao Z. (2018). Corporate culture, environmental innovation and financial performance. *Business Strategy and the Environment*.

[14] Martins J., Abreu A., Calado J. (2019). *The Need to Develop a Corporate Culture of Innovation in a Globalization Context*.

[15] Boubakri N., Chkir I., Saadi S., Zhu H. (2020). Does national culture affect corporate innovation? International evidence. *Journal of Corporate Finance*.

[16] Peri S. (2020). Enabling innovation: organizational culture and structure to the fore. *NHRD Network Journal*.

[17] Rarenko A. A., Kuo S. R., Chien C. T. (2019). *On the Technology of Assessing the Corporate Culture of Innovation Enterprises*.

[18] Shanmuganathan A. (2018). Innovation culture a part of corporate dna. *Australian Journal of Experimental Agriculture*.

[19] Turro A., Urbano D., Peris-Ortiz M. (2020). Culture and innovation: the moderating effect of cultural values on corporate entrepreneurship. *Technological Forecasting and Social Change*.

[20] Viltard R. D. L. A., Acebo M. N. (2018). Corporate culture: a key to stimulate innovation. *Independent Journal of Management & Production*.

[21] Wang Y., Farag H., Ahmad W. (2021). Corporate culture and innovation: a tale from an emerging market. *British Journal of Management*.

[22] Wu Y., Dong B. (2021). Independent director network and corporate innovation: evidence from a natural experiment in China. *Applied Economics Letters, Taylor & Francis Journals*.

